# A Novel Molecular Representation Learning for Molecular Property Prediction with a Multiple SMILES-Based Augmentation

**DOI:** 10.1155/2022/8464452

**Published:** 2022-01-28

**Authors:** Chunyan Li, Jihua Feng, Shihu Liu, Junfeng Yao

**Affiliations:** ^1^Yunnan Minzu University, Kunming, China; ^2^School of Informatics, Xiamen University, Xiamen, China

## Abstract

Deep learning has brought a rapid development in the aspect of molecular representation for various tasks, such as molecular property prediction. The prediction of molecular properties is a crucial task in the field of drug discovery for finding specific drugs with good pharmacological activity and pharmacokinetic properties. SMILES string is always used as a kind of character approach in deep neural network models, inspired by natural language processing techniques. However, the deep learning models are hindered by the nonunique nature of the SMILES string. To efficiently learn molecular features along all message paths, in this paper we encode multiple SMILES for every molecule as an automated data augmentation for the prediction of molecular properties, which alleviates the overfitting problem caused by the small amount of data in the datasets of molecular property prediction. As a result, by using the multiple SMILES-based augmentation, we obtained better molecular representation and showed superior performance in the tasks of predicting molecular properties.

## 1. Introduction

Traditionally, drug discovery is time-consuming and very expensive. For understanding the properties of a compound, many results of the simulations can be obtained via the experience of a chemist or pharmacist. The overall process is significantly complex, long, and always inefficient. Deep learning has brought a rapid development in the field of drug discovery and is expected to accelerate the process of drug discovery [1–8]. Nevertheless, deep learning methods still face some obstacles, such as small amount of data in molecular datasets, few label data [3], and label noise [5, 6], which leads to overfitting and poor model prediction performance.

Inspired by natural language processing techniques, many deep learning models use the simplified molecular input line entry system (SMILES) [9] as a line text representation of a molecule. SMILES string is in form of a 1D sequence of chemical structure that can be encoded using a one-hot vectorization form. A molecule may have multiple SMILES. Because SMILES are not unique, a molecule is often defined by canonical SMILES [10], which ensures that each molecule corresponds to a unique canonical SMILES. The SMILES-based methods [11–16] have shown great potential and have been widely used in the tasks of molecular property prediction [12–14] and molecular generation [15, 16]. The performances of the deep learning models are hindered by the nonunique nature of SMILES string, which affects the accuracy of molecular property prediction and the ability to explore the potential chemical space of molecules in molecular generation tasks [11]. Paul et al. proposed a mixed deep learning network architecture CheMixNet [12] to learn molecular representation by using several neural networks design (convolutional neural network (CNN), recurrent neural network (RNN), and multilayer perceptron (MLP)) for learning molecular SMILES sequences and molecular ACCess (MACCS) fingerprints, respectively. Then, concatenate the two parts of features and make the final prediction. Lin et al. learn molecular representation by using bidirectional gated recurrent unit (BiGRU) neural network architecture based on sequence manner [13], which is designed for solving the single- and multitask classification in the field of drug discovery. The methods input single SMILES sequence for a molecule to neural networks to learn representation. Therefore, the limited molecular representation affects the predictive performance of the neural network models. SMILES2vec [14] was proposed to train on SMILES for predicting chemical property using an RNN neural network via Bayesian optimization methods [17]. SMILES2vec was inspired by language translation using RNN in the field of natural language processing (NLP). SMILES2vec did not explicitly encode the grammar of SMILES specification. The LSTM-based [18] or GRU-based [19] recurrent neural network architecture is an effective neural network design for learning features from sequence or text data. The above neural network models based on SMILES have limitations because only the single SMILES of each molecule is considered, which cannot learn the grammatical features of SMILES well. Although SMILES enumeration [11] and all SMILES variational autoencoder [15] have considered multiple SMILES strings of single molecule to learn latent molecular representation. However, these methods are not used in the tasks of molecular property prediction. In this paper, we proposed a novel molecular representation method for molecular property prediction using multiple SMILES-based augmentation to alleviate the problem of a small amount of data and few labels in the molecular property prediction datasets， regardless of descriptors engineering and expert experience.

## 2. Related Work

A related method to this paper is the SMILES enumeration [11]. SMILES enumeration explored the fact that multiple SMILES represent the same molecule as a technique for data augmentation. The augmented dataset was bigger than the original. The neural network trained with the augmented dataset showed better performance on the test set than the original neural model trained with the unaugmented dataset. Another SMILES enumeration-based method is all SMILES variational autoencoder [15], which used multiple SMILES strings of single molecule to learn latent molecular representation for molecular generation. All SMILES variational autoencoder (VAE) encoded multiple SMILES by using several recurrent neural network layers and decoded them to molecular SMILES. All SMILES VAE learned a bijective mapping between molecules and the latent representations near the high-probability subspace of the prior. The result showed that all SMILES VAE obtained the state-of-the-art performance. However, these methods are not used in the tasks of molecular property prediction, recommended by MoleculeNet [8].

## 3. Methods

The key idea is that we focus on a multiple-SMILES representation learning as data augmentation for various downstream tasks. As we all know, the deep learning model must be fed with a large amount of data. Through learning a large amount of data, the model can find the law and obtain the potential knowledge of the data. Despite the presence of a large number of molecules, labeled datasets are scarce. In the task of molecular property prediction, the number of molecules in some datasets of property prediction is also very small. It leads to the problem of unstable prediction performance using the deep learning models due to overfitting and underfitting.

Inspired by the SMILES enumeration [11] and all SMILES VAE [15], we proposed a novel method of molecular property prediction using multiple SMILES-based augmentation to solve the overfitting and underfitting problem. The general framework is illustrated in Figure 1. Generally, before feeding the data into the deep neural network, the multiple SMILES-based augmentation must be completed (Figure 1(a)), which is related to whether the model can learn the potential knowledge in the datasets. It is a crucial step for the successful prediction of deep neural model. The process of data augmentation includes cleaning data and removing invalid molecules. Then multiple SMILES sequences are generated for each molecule, and further one-hot vectorization is carried out that can be fed to the neural network to learn molecular features. The deep neural network used in this paper is shown in Figure 1(b), which consists of stacked CNN and RNN. The “Gate” in Figure 1(b) is denoted as the gated recurrent unit (GRU) or long-short-term memory (LSTM). The final molecular representation can be used for a variety of downstream tasks, such as molecular property prediction.

In the following, we will describe technical details. We first give the mathematical definition of the problem (Section 3.1) and then propose a novel molecular representation method using multiple SMILES-based augmentation for molecular property prediction (Section 3.2).

### 3.1. Problem Definition

We define a feed-forward convolutional neural network as *𝒞𝒩𝒩*_(kernel,channel,padding)_, where kernel is the convolution kernel, channel denotes the convolution channel, and padding represents the type of padding. A recurrent neural network can be defined as ℛ*𝒩𝒩*_gate_, where gate denotes the type of gate, such as LSTM and GRU. Let *X*_*os*_ be the original SMILES strings that have been cleaned and are valid molecules. Let mapping function of multiple SMILES be *f*_*ms*_. *X*_*ms*_ is the multiple SMILES sequences. We define the vectorization function as *f*_vect_. The problem is to learn the function *f*_res_ that maps the multiple SMILES vectors to molecular representation *X*_mol_. The mapping relations are represented as follows:

(1) $$\begin{array}{c} X_{ms}=f_{ms}\left(X_{os}\right),\\ \left[f_{\text{vect}}\left(X_{ms}\right);CNN_{\left(\text{kernel,channel,padding}\right)},ℛNN_{\text{gate}}\right]\overset{f_{\text{res}}}{⟶}\;X_{\text{mol}}. \end{array}$$

The whole process includes three mapping functions, namely, *f*_*ms*_, *f*_vect_, and *f*_res_. The final molecular representation is what we want to get and can be further used in specific tasks such as molecular property prediction.

### 3.2. Multiple SMILES-Based Augmentation

The SMILES [9] is a popular specification for extracting the feature of molecular sequences that uses ASCII strings encoding molecular structures in the form of a line notation. The SMILES structure follows a certain grammar. The alphabets and numbers in SMILES denote atoms and rings, respectively. The special characters such as “=” and “≡” indicate the bond types, and the parentheses indicate side chains. The mapping function of multiple SMILES *f*_*ms*_ can be implemented using the method of renumbering atoms in RDKit [20] after performing randomization of a SMILES sequence and then regenerating a new SMILES sequence using the “MolToSmiles” method and setting canonical to be “False” in RDKit.  Figure 2 takes estradiol as an example to randomly generate 10 multiple SMILES sequences. Estradiol is randomly selected from the ESOL dataset.  Figure 3 demonstrates randomly generated 4 SMILES sequences with renumbered atoms in the molecular graph for estradiol. It is shown that atoms with different numbers in the molecule can generate different SMILES sequences. Therefore, the SMILES sequence of molecules is not unique, but canonical SMILES are unique for specific molecule.

The mapping function *f*_*vect*_ can be implemented using language translation technology in the field of natural language processing, which is an effective method for learning from text data. We need to construct a character set for all SMILES sequences in some datasets, which is similar to the corpus in natural language processing. Then randomization and vectorization to convert the SMILES array to a one-hot vector are performed.  Figure 4 demonstrates the one-hot images of vectorization using multiple SMILES for estradiol. Each image of vectorization in Figure 4 highlights the one-hot vector for different SMILES sequences. The abscissa interval is [0, 9], and the 9 represents the number of characters contained in the character set. The interval of the ordinate is [0, 37], and the 37 denotes the length of the SMILES string (including predefined extra padding).

The last mapping function *f*_res_ for obtaining molecular representation can be learned using stacked CNN and RNN mixed architecture. The RNN consists of an input layer, a hidden layer, and an output layer.  Figure 5 shows the simple structure of RNN, where *X* is an input vector, *H* indicates the hidden vector of the hidden layer, *O* represents the output vector. *W*_*xh*_,  *W*_*ho*_, and *W*_*h*_ denote the weight matrix from input layer to hidden layer from hidden layer to output layer, and hidden layer, respectively.

Figure 6 demonstrates the timeline structure of RNN. The output *O*_*t*_ of RNN at time *t* is related not only to the input *x*_*t*_ at time *t* but also to the hidden layer value *h*_*t*−1_ at time *t* − 1. It is shown that RNN can better deal with sequence information, that is, the previous input is related to the subsequent input. SMILES string is precisely this sequence structure, which can extract features with designed RNN architecture.

The message passing process for stacked CNN and RNN mixed architecture can be found in Figure 7, which shows the message passing in the neural network at time *t* and time *t* − 1. The result of the output layer at time *t* must be based on the input at time *t* and the result vector of the hidden layer at time *t* − 1. The process can be summarized in the form of matrix as follows:

(2) $$\begin{array}{c} O_{t}=P\left(W_{\text{ho}}\cdot H_{t}\right),\\ H_{t}=Q\left(W_{xh}\cdot X_{t}+W_{h}\cdot H_{t-1}\right), \end{array}$$

where *𝒫* and 𝒬 indicate some kind of neural network. Finally, the mapping function *f*_res_ for obtaining molecular representation can be represented using CNN and RNN as follows:

(3) $$\begin{array}{c} X_{cnn}=\;CNN_{\left(\text{kernel,channel,padding}\right)}\;\left(f_{\text{vect}}\left(X_{ms}\right)\right),\\ O_{t}=ℛNN_{\text{gate}}\left(W_{ho}\cdot \left(Q\;\left(W_{xh}\cdot X_{cnn}^{\left(t\right)}+W_{h}\cdot H^{\left(t-1\right)}\right)\right)\right),\\ X_{\text{mol}}=f_{\left(\text{Dense,Pooling,Gather}\right)}\left(O_{t}\right), \end{array}$$

where *f*_(Dense,Pooling,Gather)_ denotes the mapping of full-connection layer, pooling layer, and gather layer.

## 4. Experiments

Extensive experiments have been implemented to evaluate the performance of molecular representation using the multiple SMILES-based augmentation for the tasks of molecular property prediction. We will describe the datasets, baselines, and experimental results.

### 4.1. Dataset Description

We use five molecular property datasets recommended by MoleculeNet [8] for the experiments.  Table 1 shows the information of five datasets.

The details of used datasets are shown as follows:

- ESOL: ESOL [22] contains the logarithmic aqueous solubility (mol/L) of 1,127 compounds, which is used as a regression task to predict water solubility in deep neural networks
- Lipophilicity: lipophilicity [23] includes the octanol/water distribution coefficient (logD at pH 7.4) about 4,200 compounds, which is important in membrane permeability and solubility
- FreeSolv: FreeSolv [24] provides the hydration free energy (kcal/mol) of 642 compounds in water
- HIV: HIV [25] is used as a classification task in deep neural networks to predict the activity of inhibiting HIV replication, which contains 41,127 compounds
- BACE: BACE [26] is used as a classification task, which contains 1,513 molecules and provides quantitative and qualitative binding results for a set of inhibitors

The datasets must be cleaned before being input into the neural network. The cleaning and preprocessing process are shown in Figure 8. The original data are cleaned via five steps, namely, excluding invalid molecules, filtering organic molecules, removing salt and stereochemistry information, keeping the largest fragment, and converting to canonical SMILES. Then, we get the cleaned molecules that will be used to generate multiple SMILES sequences and vectorization. Finally, the feature of vectorization will be fed to the neural network to be trained.

### 4.2. Baselines

We compared our method with the following models:

1. CheMixNet: CheMixNet [12] was proposed for predicting chemical properties using molecular SMILES sequences and fingerprints, which is a mixed deep neural network architecture. In this paper, we focus on the molecular SMILES sequence. Therefore, we do not consider computable characteristics, such as molecular fingerprints or physical descriptors. For a fair comparison with our method, we adopt the neural architecture of CNN and RNN in CheMixNet [12], which uses the SMILES as the sole input.
2. Smi2Vec-BiGRU: Smi2Vec + BiGRU [13] was proposed for learning atoms and the single- and multitask classification tasks, which learns the low-dimensional representation for a molecule by transforming SMILES to vector based on bidirectional gated recurrent unit (GRU) [18] architectures.
3. XGBoost: XGBoost [27] is an ensemble method to implement a gradient boosting decision tree (GBDT) for improving the speed and efficiency of the model.
4. Multitask: Multitask network [28] was proposed for sharing the processed input among all learning tasks in a dataset and then used separate linear classifiers or regressors for each different task.
5. MPNN: Message Passing Neural Network (MPNN) is a generalized graph-based architecture [29], including the message passing phase and readout phase. The former phase is to learn the characteristics of the graph, and the latter phase is to obtain the full graph representation for predicting various tasks.
6. GC: GC [30] is a standard feature extraction method for molecules based on circular fingerprints, which is a kind of graph convolutional model and operates directly on graphs with arbitrary size and shape.
7. Weave: Weave [31] implemented graph convolutional operation on molecules using a simple encoding of the molecular graph including atoms, bonds, and distances.
8. Pretraining GNN: pretraining GNN [32] proposed a new strategy and self-supervised methods for pretraining graph neural networks. In order to obtain useful local and global features, the strategy of pretraining GNN is to pretrain expressive graph neural networks by using individual nodes and entire graphs. Pretraining GNN achieved state-of-the-art performance on the tasks of molecular property prediction.
9. Drug3D-Net: Drug3D-Net [2] is a grid-based 3D model for molecular representation using spatial-temporal gated attention, which uses the geometric information of molecules to extract the molecular characteristics.
10. Multiple SMILES (RNN (one layer), RNN (two layers), CNN_RNN): this is the method presented in this article. The neural network architecture includes one layer RNN, two layers RNN, and the mixed networks of CNN and RNN.

### 4.3. Experimental Setup

In this experiment, we use root mean squared error (RMSE) and mean absolute error (MAE) to evaluate the performance of regression tasks. Similarly, we use the loss function of “binary_crossentropy” for classification datasets. We use the average area under the receiver operating characteristics curve (AUROC) and the area under the precision-recall curve (AUPRC) predicted from the test set to evaluate the performance of the model for classification tasks. Our experiment was trained based on the Keras framework and TensorFlow [33]. We used the Adam algorithm [34] for optimizing the parameters of the model. We set a total of 200 epochs, 64 batch sizes, and 5-fold cross-validation with checkpoint and early stopping. We set the learning rate as 0.001 with learning rate decay. We perform randomization of a SMILES string with the random number 5 for ESOL, lipophilicity, FreeSolv, and BACE datasets. As for the HIV dataset, we set random number 20 to implement multiple SMILES randomization only for positive samples so that we obtain a total of 30,303 positive examples compared with the original 39,684 negative samples.

### 4.4. Performance Comparison

#### 4.4.1. Performance in Regressions

Solubility, lipophilicity, and free energy are very important physical chemistry properties, which are essential properties to understand molecular interaction with solvents.  Table 2 demonstrates the predictive performances for water solubility (ESOL), octanol/water distribution coefficient (lipophilicity), and hydration free energy (FreeSolv). Our multiple SMILES-based model using mixed CNN and RNN architecture obtains the best performance. The smaller the value of RMSE and MAE, the better for ESOL, lipophilicity, and FreeSolv. As shown in Table 2, we obtain 0.4448 MAE and 0.5916 RMSE values for ESOL in the test set. The RMSE value of 0.5916 is slightly lower than the MPNN with the 0.5800 RMSE. However, as for lipophilicity and FreeSolv datasets, our method obtains superior performance on both RMSE and MAE values, which shows that the multiple SMILES-based data augmentation can alleviate the overfitting problem to a certain extent on a small amount of data, such as ESOL and FreeSolv datasets.

Figure 9 shows the scatter plots in the FreeSolv dataset for four training-folds, which indicates that the points on the test set closely surround the identity line, which shows that the prediction results in the test set are closer to the target value, although the trend lines deviate slightly from the identity lines in each training folds. In addition, Figure 10 shows the loss curves during our model training in the training set and validation set for the FreeSolv dataset. At the beginning of the training of the model, the loss on the training set and the validation set has a relatively large gap (training loss curve and validated loss curve are far away), indicating that the model is not stable. When the number of training epochs increases, the loss curves on the training set and the validation set tends to be consistent and fit each other, indicating that the model tends to be stable and is slowly converging.

#### 4.4.2. Performance in Classifications

Table 3 demonstrates the predictive performances for HIV activity (HIV) and inhibitors of human *β*-secretase 1 (BACE). The larger the AUROC and AUPRC score, the better for HIV and BACE. Our method based on mixed CNN and RNN architecture achieved the best performance on AUROC and AUPRC scores in the test set for HIV and BACE datasets. In HIV, we obtain 0.9767 AUROC and 0.9798 AUPRC scores compared with the 0.9621AUROC and 0.9617 AUPRC of the 3D-based method Drug3D-Net, although the Drug3D-Net considered the information of molecular geometry. In addition, the performance of our method exceeds that of the pretrained model pretraining GNN with a large margin.

In summary, our method shows superior performance in both regression datasets and classification datasets, which implies the good molecular representation ability of our proposed method.

### 4.5. Ablation Study

For different neural architectures of our multiple SMILES methods (shown in Tables 2 and 3), the mixed CNN_RNN architecture obtains the best performance among RNN (one layer), RNN (two layers), and CNN_RNN, which indicates that the CNN convolution in our model is essential and can improve the predictive performance for downstream tasks. Meanwhile, the performance of RNN (two layers) architecture is slightly better than that of RNN (one layer) architecture, which shows that the deeper neural networks can have better learning ability for extracting features. Therefore, it can show better performance in specific tasks, such as molecular property prediction.

## 5. Conclusion

In this study, we make full use of the nonunique nature of the SMILES string to perform randomization of a SMILES string multiple times for efficiently learning molecular features along all message paths. By encoding multiple SMILES for every molecule as an automated data augmentation, we obtain better molecular representation and the proposed method shows superior performance in the tasks of predicting molecular properties, which alleviates the overfitting problem caused by the small amount of data in the datasets of molecular property prediction.

## Figures and Tables

**Figure 1:** The architecture of molecular representation with a multiple SMILES-based augmentation for molecular property prediction. (a) The process of data augmentation using multiple SMILES. After cleaning and removing invalid molecules from the original datasets, multiple SMILES sequences are generated for each molecule, and further one-hot vectorization is carried out. (b) The stacked CNN and RNN neural networks. After passing through different layers (including dense layer, dropout layer, pooling layer, and gather layer), finally the characteristics such as molecular properties are predicted.

**Figure 2:** The generation of multiple SMILES for estradiol. The original SMILES is “CC12CCC3C(CCc4cc(O)ccc34)C2CCC1O” that is randomly selected from the ESOL dataset. Here, it is shown the randomly generated 10 SMILES sequences for estradiol molecule.

**Figure 3:** The randomly generated 4 SMILES sequences with renumbered atoms in the molecular graph for estradiol.

**Figure 4:** The images of one-hot vectorization using multiple SMILES for Estradiol molecule. It shows the vectorization of randomly generated 6 SMILES strings, using random order of the character set for Estradiol, which consists of 9 characters: “(”, “3”, “O”, “c”, “1”, “)”, “2”, “4”, “C”. The length of padding is 37, that includes predefined extra padding. (a) c12cc(O)ccc1C1C(C3CCC(O)C3(C)CC1)CC2. (b) C1(O)C2(C)C(CC1)C1C(c3c(cc(O)cc3)CC1)CC2. (c) C12(C)C(CCC1O)C1C(c3ccc(O)cc3CC1)CC2. (d) Oc1ccc2c(c1)CCC1C3CCC(O)C3(C)CCC12. (e) OC1C2(C)CCC3c4ccc(O)cc4CCC3C2CC1. (f) C1C2c3ccc(O)cc3CCC2C2CCC(O)C2(C)C1.

**Figure 5:** The structure of the recurrent neural network [21].

**Figure 6:** The timeline structure of the recurrent neural network [21].

**Figure 7:** The message passing process for stacked CNN and RNN.

**Figure 8:** The process of data cleaning and preprocessing.

**Figure 9:** Scatter diagram of FreeSolv dataset for four training folds. The horizontal axis is the ground truth value, and the vertical axis is the predicted value by our model. The solid lines indicate the trend lines, and the dashed lines indicate the identity lines. The blue and red points represent the predicted values in the validation set and test set, respectively.

**Figure 10:** The loss curves during our model training for FreeSolv in the training set and validation set.

**Table 1:** The description of public molecular datasets, including data type, task type, and the number of compounds before and after augmentation.

Dataset	Data type	Task type	Compound	Compound after augmentation
ESOL	SMILES	Regression	1127	6762
Lipophilicity	SMILES	Regression	4200	25200
FreeSolv	SMILES	Regression	642	3852
HIV	SMILES	Classification	41127	69987
BACE	SMILES	Classification	1513	9078

**Table 2:** The RMSE and MAE values of various approaches in ESOL, lipophilicity, and FreeSolv datasets. The predictive values of the approaches are partly derived from the related references [2, 8].

Model		ESOL		Lipophilicity		FreeSolv	
		RMSE	MAE	RMSE	MAE	RMSE	MAE
CheMixNet	CNN_RNN	1.0419	0.8010	1.0513	0.8282	1.3553	1.0156

Conventional methods	XGBoost	0.9900	—	0.7990	—	1.7400	—
	Multitask	1.1200	—	0.8590	—	1.8700	—

Graph-based methods	MPNN	**0.5800**	—	0.7190	—	1.1500	—
	Weave	0.6100	—	0.7150	—	1.2200	—

3D-based models	Drug3D-Net	0.9683	0.7841	0.9930	0.8404	1.4709	1.1598

Our method (multiple SMILES)	RNN (one layer)	0.6585	0.5105	0.7929	0.6211	1.6051	1.2313
	RNN (two layers)	0.6394	0.4940	0.7960	0.6217	1.3575	1.0468
	CNN_RNN	0.5916	**0.4448**	**0.7054**	**0.5481**	**1.0033**	**0.7859**

The best results are highlighted in bold.

**Table 3:** The AUROC and AUPRC scores of various approaches in HIV and BACE datasets. The predictive values of the approaches are partly derived from the related references [2, 8, 13, 32].

Model		HIV		BACE	
		AUROC	AUPRC	AUROC	AUPRC
CheMixNet	CNN_RNN	0.8204	0.8614	0.7429	0.7162

SMILES-based	Smi2Vec-BiGRU	0.9117	0.8963	0.8440	0.7872

Conventional methods	XGBoost	0.7560	—	0.8500	—
	Multitask	0.6980	—	0.8240	—

Graph-based methods	GC	0.7630	—	0.7830	—
	Weave	0.7030	—	0.8060	—
	Pretraining GNN	0.7990	0.7806	0.8450	0.7908

3D-based models	Drug3D-Net	0.9621	0.9617	0.7185	0.6397

Our method (multiple SMILES)	RNN (one layer)	0.9567	0.9525	0.7879	0.7577
	RNN (two layers)	0.9613	0.9636	0.8083	0.7665
	CNN_RNN	**0.9767**	**0.9798**	**0.8512**	**0.7919**

The best results are highlighted in bold.

## Data Availability

All input data are publicly available and a detailed description for the same is mentioned in the Dataset Description.
